The article "Application of Internet of Things on the Healthcare Field Using Convolutional Neural Network Processing" was published in 2022. Journal: J Healthc Eng.

# Application of Internet of Things on the Healthcare Field Using Convolutional Neural Network Processing

**DOI:** 10.1155/2022/1892123

**Published:** 2022-01-25

**Authors:** J. Mohana, Bhaskarrao Yakkala, S. Vimalnath, P. M. Benson Mansingh, N. Yuvaraj, K. Srihari, G. Sasikala, V. Mahalakshmi, R. Yasir Abdullah, Venkatesa Prabhu Sundramurthy

**Affiliations:** ^1^Department of Electronics and Communication Engineering, Saveetha School of Engineering, SIMATS, Chennai, Tamil Nadu, India; ^2^Department of Electronics and Communication Engineering, Erode Sengunthar Engineering College, Erode, Tamil Nadu, India; ^3^Department of Electronics and Communication Engineering, Sri Ramakrishna Institute of Technology, Coimbatore, Tamil Nadu, India; ^4^Research and Publications, ICT Academy, IIT Madras Research Park, Chennai, Tamil Nadu, India; ^5^Department of Computer Science and Engineering, SNS College of Technology, Coimbatore, Tamil Nadu, India; ^6^Department of Electronics and Communication Engineering, Vel Tech Rangarajan Dr. Sagunthala R&D Institute of Science and Technology, 400 Feet Outer Ring Road,Avadi, Chennai 600062, Tamil Nadu, India; ^7^CSBS, Sri Krishna College of Engineering and Technology, Coimbatore, Tamil Nadu, India; ^8^Center of Excellence for Bioprocess and Biotechnology, Department of Chemical Engineering, College of Biological and Chemical Engineering, Addis Ababa Science and Technology University, Addis Ababa, Ethiopia

## Abstract

Population at risk can benefit greatly from remote health monitoring because it allows for early detection and treatment. Because of recent advances in Internet-of-Things (IoT) paradigms, such monitoring systems are now available everywhere. Due to the essential nature of the patients being monitored, these systems demand a high level of quality in aspects such as availability and accuracy. In health applications, where a lot of data are accessible, deep learning algorithms have the potential to perform well. In this paper, we develop a deep learning architecture called the convolutional neural network (CNN), which we examine in this study to see if it can be implemented. The study uses the IoT system with a centralised cloud server, where it is considered as an ideal input data acquisition module. The study uses cloud computing resources by distributing CNN operations to the servers with outsourced fitness functions to be performed at the edge. The results of the simulation show that the proposed method achieves a higher rate of classifying the input instances from the data acquisition tools than other methods. From the results, it is seen that the proposed CNN achieves an average accurate rate of 99.6% on training datasets and 86.3% on testing datasets.

## 1. Introduction

Data collection has become much easier, thanks to the rise of smart Internet-of-Things (IoT) devices and sensors. However, the analysis and utilization of data still face challenges associated with incorrect feature extraction. When faced with these difficulties, researchers and specialists began looking for optimal solutions that allow extraction of most possible data from a given dataset. Our ability to learn more about our surroundings has improved since the invention of AI in the late twentieth century.

Ongoing advancements in artificial intelligence (AI) have been implemented in numerous industries, including the education and medical field. According to numerous studies [1–3], AI has shown the ability to outperform humans and information systems at most cases [4–8]. It is a mechanical, electrical, and chemical organism that constitutes the human body [5]. Electrocardiogram (ECG) signals are a biophysical indicator of the electrical activity of the heart. It shows how the beating of the heart changes over time [9–13]. Automated systems have a difficult time spotting anomaly. External noise and the body response to different physical conditions are examples of this [6–8].

To our knowledge, convolutional neural network (CNN) works well with ECG recordings from the data acquisition IoT devices. Appropriate ECG signal processing with the CNN learns features using patient needs with abnormalities in arrhythmia and heart failure [14–16].

In this paper, we develop the convolutional neural network (CNN) architecture, which we examine in this study to see if it can be implemented. The study uses the IoT system with a centralised cloud server, where it is considered as an ideal input data acquisition module.

The main contribution of the work involves the following:

- The authors develop a sparse CNN with autoencoding properties in order to improve the accuracy of classification.
- The speed and reliability of IoT systems are heavily dependent on the speed and reliability of the internet connection used. Smart gateway devices lack the processing power to execute CNN methodologies.
- The study uses cloud computing resources by distributing CNN operations to the servers with outsourced fitness functions to be performed at the edge. It is therefore enabling improved system availability by making decisions at the local level.
- An ECG classification using input IoT data acquisition modules is evaluated in terms of response time and accuracy in a real-world case study.

## 2. Background

Each of the six waves in the ECG waveform is separated into two waves, two segments, and one complicated wave. During the initial electrical activity of the human heart, which is known as the PR interval, the right atrium chamber depolarizes, causing deoxygenated blood to exit via the vena cava into the right ventricle. It is at this point that two distinct pumping mechanisms kick into high gear: one to move deoxygenated blood to the lungs for oxygenation and the other to move oxygenated blood throughout the remaining part of the body. To begin another heartbeat cycle, the heart ventricles must be repolarized during the QT interval including the QRS complex, the ST segment, and the *T*-wave.

Some of the most critical and subtle ECG signals may be missed by commonly used applications that only count the number of beats per second and ignore the ECG signal pattern morphology that changes without altering the cycle normal time. A great deal of effort has gone into figuring out how to get useful information out of such sensitive medical records. Several methods utilizing the feature extraction based on features, feature combinations, or a selection of features were presented [17]. Time-frequency analysis of ECG signals can be done using wavelet transforms developed by the authors in [18]. In this paper, ECG classification using a CNN is presented to address these shortcomings. CNNs are a type of hierarchical artificial neural networks (ANNs) [19, 20] that use downsampling and convolutional layers to alternately mimic the human visual cortex cells.

## 3. Proposed Method

Figure 1 shows an autoencoder with the hidden layer for learning features from the input *x* if there are data *x*={*x*_1_, *x*_2_, *x*_3_, *x*_4_, *x*_5_} available. All three layers are referred to as input, hidden, or reconstitution layers. The input layers are connected directly with layer 2 or hidden layers, where it performs various operations of autoencoding, and then layer 3 performs the process of providing the outputs of the hidden layers.

The goal of the reconstitution layer is to minimize the error between the layers. The hidden layer can be thought of as a different way to represent data because the essential characteristics of the data can be extracted from it.

Autoencoder networks are actually designed to learn the activation function *h*_*W*,*b*_(*x*) ≈ *x*. The limited neurons in the hidden layer extract the hidden features. As an example, 1024 neurons can be used to process a 32 × 32 matrix image. In a similar way to PCA and other dimension reduction methods, this is what this does. However, the hidden layer contains only a few neurons. According to this constraint, any network can be made to become sparse if the activation value of each hidden layer *j*^th^ neuron is *a*_*j*_.

(1) $$\begin{array}{c} \rho_{j}=\frac{1}{m}\sum_{i=1}^{m}a_{j}x_{i}, \end{array}$$

where *m* is the input layer neurons and *ρ*_*j*_ is the sparse constraint constant (like 0.05).

The study uses the KL distance function to optimise *ρ*_*j*_ when solving the hidden layer.

(2) $$\begin{array}{c} \text{KL}\left(\rho \left\|\right)\rho_{j}\right)=\rho \;\log\frac{\rho }{\rho_{j}}+\left(1-\rho \right)\log\frac{1-\rho }{1-\rho_{j}}. \end{array}$$

CNNs use a spatiotemporal convolution kernel to specify the feature map in their convolution layer. Each feature map output of the last subsampling layer *l* consists of the bias term *b*_*j*_^*ℓ*^ and convolution kernel *W*_*ij*_^*ℓ*^ only if there exist input feature maps *N*_*in*_. The formula for estimating the feature map *X*_*j*_^*ℓ*^ of output *j* is as follows:

(3) $$\begin{array}{c} X_{j}^{\ell }=f\left(\sum_{i=1}^{N_{in}}\alpha_{ij}\left(X_{i}^{\ell -1}*W_{ij}^{\ell }\right)+b_{j}^{\ell }\right). \end{array}$$

Additionally, it must adhere to the following rules:

(4) $$\begin{array}{c} \sum_{i}\alpha_{ij}=1,\\ 0\leq \alpha_{ij}\leq 1. \end{array}$$

Backpropagation begins with determining how each subsampling layer (*l*) is connected to its next convolution layer, and this must be done before we can begin the process, so as to conduct backward the next layer residual *δ*^*ℓ*+1^. To determine the feature map of the *j*^th^ residual (*δ*_*j*_^*ℓ*^) layer, we can apply the gradient descent method. Suppose the layer activation function *f* which is the derivative of *f*′(*z*_*j*_^*ℓ*^) has the input *z*_*j*_^*ℓ*^. The formula for the calculation is as follows:

(5) $$\begin{array}{c} \delta_{j}^{\ell }=f{}^{\prime }\left(z_{j}^{\ell }\right)\cdot \text{conv}2\left(\delta_{j}^{\ell +1},\text{rot}180\left(W_{j}^{\ell +1}\right)\right). \end{array}$$

In the above process, the convolution kernel conv2(·) must be rotated in order to perform cross-correlation calculations.

The sparse constraint is imposed on the output of the sparse autoencoder neural network. However, in this case, the input is limited to a sparse set of values. These two modes of operation are distinct, but they accomplish the same thing. Features can be extracted from input data using sparse autoencoder neural networks. Spatiotemporal convolution is a major change in this framework because all of the previous layer input feature maps are used as inputs for each output feature map. Due to the sparse constraints, the feature maps can be fed to the output map, and this is limited extremely.

### 3.1. Event Recognition Using the CNN

In the above framework, we feed the CNN seven consecutive 64 × 64-pixel frames in order to capture ECG data encoded in the input image frame, with the current image frame serving as the centre of attention. Assume that each frame in the input set is a 64 × 64 greyscale image with the same dimensions. Scaling is required if the dimensions are different from one another.

Convolution kernels of the form 7 × 5 × 5 can be used by the C1 layer to obtain 36 feature maps to extract 36 different features from the input frames. As complicated as action event classification is, the 36 feature maps are perfectly capable of classifying the simple action. On the contrary, the convolution kernel is 5 × 5 in the space dimension. In other words, each C1 layer feature map is linked to all seven 5 × 5 image blocks. The C1 layer produces 36 number of 60 × 60-pixel feature maps as a result.

It is a sampling layer, the S1 layer. Accordingly, the C1 layer feature maps are rescaled to improve the CNN resilience to scale changes and minor deformations. The subsampling layer scaling factor cannot be too large.

## 4. Results and Discussion

In this section, the entire simulation is conducted in the Python environment to study the effectiveness of the proposed model.  Table 1 shows the proposed CNN which is compared with existing image classification models such as VGG-16, ResNet-50, Inception V3, EfficientNetB0, and EfficientNetB7, the parameters of which are given in Table 1.

The proposed CNN is compared with existing methods such as VGG-16, ResNet-50, Inception V3, EfficientNetB0, and EfficientNetB7 in terms of various performance metrics including accuracy, precision, recall, *F*-measure, and percentage error. Moreover, the running time of the proposed method is tested on training and testing times.

Table 2 shows the results of accuracy between the proposed CNN and existing methods such as VGG-16, ResNet-50, Inception V3, EfficientNetB0, and EfficientNetB7. The results of the simulation are conducted on both training and testing stages. The results of accuracy show that, at the time of training, the study has more accuracy than at the testing stage. Moreover, it is seen that the proposed CNN has higher classification accuracy than other methods.

Table 3 shows the results of run time between the proposed CNN and existing methods such as VGG-16, ResNet-50, Inception V3, EfficientNetB0, and EfficientNetB7. The results of the simulation are conducted on both training and testing stages. The results of run time show that, at the testing stage, it has higher run time than the training stage. Moreover, it is seen that the proposed CNN has reduced run times than other methods.

Figure 2 shows the results of precision between the proposed CNN and existing methods such as VGG-16, ResNet-50, Inception V3, EfficientNetB0, and EfficientNetB7. The results of precision show that, at the time of the testing stage, the proposed CNN has higher precision rate than other methods.

Figure 3 shows the results of recall between the proposed CNN and existing methods such as VGG-16, ResNet-50, Inception V3, EfficientNetB0, and EfficientNetB7. The results of recall show that, at the time of the testing stage, the proposed CNN has higher recall rate than other methods.

Figure 4 shows the results of *F*-measure between the proposed CNN and existing methods such as VGG-16, ResNet-50, Inception V3, EfficientNetB0, and EfficientNetB7. The results of *F*-measure show that, at the time of the testing stage, the proposed CNN has higher *F*-measure rate than other methods.

Figure 5 shows the results of MAE between the proposed CNN and existing methods such as VGG-16, ResNet-50, Inception V3, EfficientNetB0, and EfficientNetB7. The results of MAE show that, at the time of the testing stage, the proposed CNN has reduced MAE than other methods.

## 5. Conclusions

In this paper, CNN examines the input signal from the IoT devices, where ECG data are classified to detect the presence of arrhythmia and heart failure from the image dataset. The classification of the dataset on two different heartbeat signals enables faster training and testing packages. The utilization of cloud resources to perform the CNN classification shows fastest classification process without lags. The simulation is conducted to test the efficacy of the CNN against ECG image datasets. The simulation shows that the proposed CNN classifies well the instances than other existing methods. The results of the simulation show an improved accuracy rate of 98% than image ECG classification models. In the future, federated learning can be used to examine the multimodal signals for the purpose of improved classification of instances in case of arrhythmia and heart failure.

## Figures and Tables

**Figure 1:** Sparse CNN of autoencoding type.

**Figure 2:** Precision.

**Figure 3:** Recall.

**Figure 4:** *F*-measure.

**Figure 5:** MAE.

**Table 1:** Deep learning parameters.

Model	Parameters
VGG-16	138 million
ResNet-50	25 million
Inception V3	24 million
EfficientNetB0	5.3 million
EfficientNetB7	66 million
Proposed CNN	60,000

**Table 2:** Accuracy (%) of training and testing.

Model	Accuracy with training datasets	Accuracy with testing datasets
VGG-16	75.0	74.5
ResNet-50	87.0	76.3
Inception V3	90.7	77.15
EfficientNetB0	93.8	78.8
EfficientNetB7	94.9	84.4
Proposed CNN	99.6	86.3

**Table 3:** Running time (ms) of training and testing.

Model	Running time with training datasets	Running time with testing datasets
VGG-16	352,628	793,412
ResNet-50	38,797	117,167
Inception V3	15,652	97,854
EfficientNetB0	10,422	79,485
EfficientNetB7	5252	43,685
Proposed CNN	4556	42,965

## Data Availability

The datasets used and/or analyzed during the current study are available from the corresponding author upon reasonable request.
